The article "Residential green space associated with the use of attention deficit hyperactivity disorder medication among Dutch children" was published in 2022. Journal: Front Psychol.

# Residential green space associated with the use of attention deficit hyperactivity disorder medication among Dutch children

**DOI:** 10.3389/fpsyg.2022.948942

**Published:** 2022-09-02

**Authors:** Sjerp de Vries, Robert Verheij

**Affiliations:** ^1^Wageningen Environmental Research, Wageningen University and Research, Wageningen, Netherlands; ^2^Cultural Geography Chairgroup, Wageningen University and Research, Wageningen, Netherlands; ^3^Netherlands Institute for Health Services Research (Nivel), Utrecht, Netherlands; ^4^Tranzo, Tilburg School of Social and Behavioral Sciences, Tilburg University, Tilburg, Netherlands

**Keywords:** residential environment, green space, children, ADHD, medication, socioeconomic status, ethnicity, registry data

## Abstract

Several studies have observed an inverse relationship between attention deficit hyperactivity disorder (ADHD)-related behavior of children, as reported by parents or teachers, and the amount of green space in their residential environment. Research using other, more objective measures to determine ADHD prevalence is scarce and could strengthen the evidence base considerably. In this study, it is investigated whether a similar beneficial association will be observed if the use of ADHD-related medication is selected as an outcome measure. More specifically, registry data from a health insurance company on the reimbursement of ADHD-related medication in 2011 were available for 248,270 children between 5 and 12 years of age. Amounts of green space within 250 and 500 m of the home address were calculated. Multilevel logistic regression analyses for the prevalence of use were conducted, including the following covariates: sex, age, urbanity of the neighborhood, neighborhood socioeconomic status (SES), and percentage of people with a non-Western migration background in the neighborhood population. Results showed that the amount of green space was inversely related to the prevalence of use of ADHD medication. Moreover, the relationship was strongest among children living in the least wealthy neighborhoods and absent among those living in the wealthiest neighborhoods. Results also show that in less wealthy neighborhoods, there is, on average, less green space available nearby: children who are likely to benefit most from nearby green space tend to have the least of it.

## Introduction

Due to increasing urbanization, daily contact with nature is becoming less common, also for children (Seltenrich, 2015). A systematic review suggests that this may have detrimental consequences for the mental health of children, especially when it comes to hyperactivity and inattention problems (Vanaken and Danckaerts, 2018). According to a recent international consensus statement, attention deficit hyperactivity disorder (ADHD) is rarely caused by a single genetic or environmental risk factor, but most cases of ADHD are caused by the combined effects of many genetic and environmental risks, each having a very small effect (Faraone et al., 2021). A lack of contact with nature might be one of them. Conversely, cross-sectional studies show beneficial associations between the amount of or access to residential green space and ADHD-related issues in children (Amoly et al., 2014; Balseviciene et al., 2014; Flouri et al., 2014; Markevych et al., 2014; Lee et al., 2019). A causal interpretation of the aforementioned cross-sectional findings is supported by an experimental study showing that a walk in a green environment improved the ability to concentrate in children diagnosed with ADHD, at least for a short time (Faber-Taylor and Kuo, 2009).

This latter result is consistent with a much larger body of experimental evidence, mainly based on research on adults, showing that contact with nature has attention-restoring and stress-reducing effects (Hartig et al., 2014; Markevych et al., 2017). Theoretically, these experiments are predominantly based on the attention restoration theory (ART) and/or the stress reduction theory (SRT). The ART states that natural environments tend to require less directed attention than built-up environments, allowing restoration of this resource when it previously has been depleted (Kaplan and Kaplan, 1989). The SRT states that because of the humankind’s evolutional history, exposure to unthreatening natural settings has immediate calming effects on stressed individuals, physiologically as well as emotionally (Ulrich, 1981). Thus, according to the two theories, contact with nature may have a calming effect on children with ADHD and increase their ability to concentrate and decrease impulsive behavior. This may be facilitated by an ample supply of opportunities for such contacts in the residential environment of the children. Nearby green space may also promote active outdoor play and burning off excess energy in the process (see, e.g., Lachowycz et al., 2012). Based on a web-based survey among parents and guardians, Faber-Taylor and Kuo (2011) concluded that children officially diagnosed with ADHD who played outside in a natural environment displayed less severe symptoms than those who played indoors or in a predominantly built-up environment.

The cross-sectional studies mentioned previously make use of ADHD-related behavior, as reported by parents or teachers [for more recent examples, see Yang et al., 2019; Dzhambov et al., 2022, looking (also) at the school environment]. On the one hand, parents and teachers offer a valuable source of information, with reports being based on direct and long-term observation of the children’s behavior. On the other hand, self-selection may occur, and reporting biases may exist, especially in medically untrained people. Confirmation of these earlier findings using a different source of information on the prevalence of ADHD will strengthen the evidence base considerably. One such source is administrative data on the use of ADHD medication. In this study, we use reimbursement data from a large health insurance company in the Netherlands. It may be noted that displaying ADHD-related behavior and the reimbursement of ADHD medication do not have a one-on-one relationship: the former does not necessarily lead to the second. The observation by its parents (or its teacher) that a child displays ADHD-related symptoms may lead them to visit their family doctor. The family doctor may or may not arrive at the conclusion that the child has ADHD and, if so, may subsequently prescribe ADHD medication, such methylphenidate (see Figure 1). In addition, health insurance data concern the reimbursements of prescribed medicines. Parents may not ask for reimbursement. However, since requesting reimbursement is in their own (financial) interest, we expect reimbursement rates to closely resemble prescription rates.

**FIGURE 1:** Conceptual model relating green space to use of ADHD medication by children.

Parents may respond differently to the display of the same type of behavior. Furthermore, to the extent that a child spends more time playing outdoors, its parents may also be confronted less with (indoor) behavior that they consider annoying or undesirable, which may lower the probability that they will bring this behavior to the attention of their family doctor. Although this is not a well-researched topic, there are studies showing cultural differences in whether or not parents consider ADHD-related behavior problematic and whether or not they will take this issue to their family doctor. In the Netherlands, parents with a non-Western migration background perceive similar ADHD-type behavior as less problematic than their autochthonous counterparts, and their children also visit healthcare professionals less often with this type of problem (Bevaart et al., 2012, 2014). Although in the Netherlands, general practitioners are formally not qualified to diagnose ADHD, they frequently do so. Such informal diagnosis is not always subsequently confirmed (or rejected) by a psychiatrist or pediatrician. This implies that there may be differences between general practitioners in how they record symptoms or diagnose the same kind of behavior. They may also differ in their prescription behavior.

## Materials and methods

The study involves a secondary data analysis, in which registry data of a Dutch health insurance company are enriched with characteristics of the residential environment at the level of individual children. The two datasets were linked by the health insurance company by means of the six-digit post code of the home address of the child, which was removed before handing the dataset over for conducting the analyses. To get approval to make use of the registry data, beforehand the privacy of the children involved had to be guaranteed. This was carried out by keeping the number of environmental characteristics small, thereby precluding the identification of an individual child due to an unique combination of values in the joined dataset.

### Attention deficit hyperactivity disorder medication

Medication data were provided by Achmea, the main Dutch health insurance company in the central part of the Netherlands at the time of the research. According to Smeets et al. (2011), the Achmea Health Database (formerly Agis) is not completely representative for the entire Dutch population but does represent the urbanized area of the Netherlands. From this database, all children between 5 and 12 years of age (in 2011) were selected, regardless of whether they had used AHDH medication or not. Only children who were insured by Achmea during the whole of 2011 and 2012 were included (*n* = 274.698). Records on reimbursements for ADHD-related medication, such as methylphenidate, were aggregated by child to determine usage in 2011 (yes/no). For children, this type of medicine [Anatomical Therapeutic Chemical (ATC) code N06BA**] is almost exclusively prescribed for AD(H)D-related symptoms. To the best of our knowledge, this type of information has not been used before in studies looking at the relationship between residential green space and ADHD among children. Although Aerts et al. (2022) did use ADHD medication prescription data, they did so for adults (and not at an individual level). In addition to age, sex, and family doctor (and home address), no background characteristics of the child were available in the Achmea Health Database.

### Residential green space

Residential greenness was assessed using two methods. The first method was to look at all green types of land use, based on a national land-use database (Hazeu et al., 2014). In this database, the dominant type of land use for each 25 × 25-m raster cell is recorded in 39 categories. Version 7 of this database (LGN7) is mainly based on data from the year 2012. Green types of land use include agricultural areas (codes: 1–6, 61, and 62), forests (codes: 11, 12, 40, and 43), nature areas (30–39, 42, and 45), and urban green areas (codes: 20, 22–24, and 28). Using the center of the six-digit post code of the residential address, the most detailed spatial identifier nationally available at that time, the percentages of green area within 250 and within 500 m were calculated. On average, in 2012, about 17 households shared the same six-digit post code, with the size of the area depending on the local population density. This green space indicator has been used before in Dutch research on green space and human health, although with larger buffer sizes (see, e.g., Maas et al., 2009; Van den Berg et al., 2010). In the current study, smaller distances were chosen because of the limited radius of action of school-aged children when it comes to autonomous outdoor play. The same two distances have been used by Amoly et al. (2014).

The second method involved the use of normalized difference vegetation index (NDVI) scores, based on satellite imagery. NDVI scores indicate the amount of green biomass present. In the present study, the average NDVI scores for 25 May and 25 July 2012 was used, two cloudless days. Originally, NDVI scores range from –1 to + 1, with scores above 0 indicating the presence of green biomass. Scores below 0 may indicate water surfaces. To avoid water and vegetation averaging each other out, the original NDVI scores were recoded: scores above 0 were multiplied by 250, and scores of 0 and below were recoded to 1. Average-recoded NDVI scores were calculated for the same two distances: 250 and 500 m. NDVI scores have also been used before in studies on green space and ADHD, although not in the Netherlands (Amoly et al., 2014; Balseviciene et al., 2014). However, we calculated the average for only those raster cells within the buffer that were identified as built-up/sealed surface area within the LGN7 land-use database. This was performed to make the two greenness indicators complementary, rather than strongly overlapping. Due to being limited to the built-up area, these average NDVI scores are considered to indicate the presence of very small green areas or natural elements, such as home gardens and street trees, within the built-up part of the environment. In this study, next to the percentage of green area, we used these average NDVI values for the built-up part of the buffers. To prevent specific combinations of the two greenness characteristics for the two buffers to be uniquely linked to a six-digit post code, and thereby compromise the privacy of clients, they were recoded into broader classes. For the percentages of green space, this were twenty 5% classes. For the two NDVI scores, these were seven classes. The two extreme classes were less than 80 and more than 130, with in between five equal-interval classes of 10 points wide each.

### Additional characteristics

In addition to the two greenness indicators, each for two buffers, several characteristics of the neighborhood in which the six-digit postcode was located were added to the environmental database. The 2012 values for these characteristics were available at Statistics Netherlands (CBS) and included the level of urbanity (five levels, based on address density), the percentage of children between 0 and 14 years of age within the population (twenty 5%-classes), the percentage of inhabitants with a non-Western migration background (twenty 5%-classes), and the average residential property value (WOZ-value) (CBS, 2016). The latter was used as an indicator of the socioeconomic status (SES) of the neighborhood. Property values were recoded into seven classes. The two extreme classes were less than € 145,000 and more than € 345,000, with in between five equal-interval classes of € 40,000 wide each. The percentage of children < 15 years was included as a covariate based on the assumption that the availability of playmates in the neighborhood might increase the likelihood of outdoor play. As mentioned before, Achmea linked the environmental data to their healthcare data by using the six-digit post code, after which this post code was removed to protect the privacy of their clients. Also, the code for the family doctor was pseudonymized by Achmea. Children who moved during 2011 or 2012 (about 10%) were excluded, as were children without a valid post code or code for the family doctor. After also removing cases with missing values on any of the variables used in the analyses, 248,270 cases were available for analysis. Due to the client base of Achmea being mainly located in the middle of the Netherlands, the sample cannot the considered representative for all Dutch children in the selected age category.

### Statistical analyses

Several children are likely to live in the same neighborhood and/or be registered with the same family doctor. Thus, the dataset has a nested structure, which calls for multilevel analyses. The first level consists of children. Neighborhood and family doctor are cross-classified: children living in the same neighborhood may be listed as patients registered with a different family doctor, and vice versa. Given the large number of possible combinations of neighborhood and family doctor, both these higher levels cannot be taken into account simultaneously. To start with, separate analyses have been performed, with either neighborhood or family doctor as the second level. Based on the first results, to be reported later on, additional analyses were only performed with neighborhood as the second level. The dependent variable was whether or not the children used ADHD medication in 2011. Therefore, logistic regression analyses were performed. Regression models were built up in several steps. In the first model, only the available covariates, at either the individual or the neighborhood level, were included in the model: age, sex (categorical), urbanity (categorical), average real estate property value (categorical), percentage of non-Western immigrants, percentage of children younger than 15 years. In the second model, one of the greenness indicators was added: the percentage of green area within either 250 or 500 m or the mean NDVI score for the built-up area within one of those distances. In the third model, both the percentage of green area and the average NDVI score for the same distance were included in the model. In a fourth step, different moderators were tested one by one, by introducing interaction terms. This was carried out for average residential property value, sex, and age. For the average residential property value, interaction terms were created by first reducing the number of categories to three, by combing the lowest two, the middle three, and the upper two categories, respectively. For age, this was performed by means of a multiplicative interaction term (with both variables centered beforehand). The multilevel analyses were performed by MLwiN, versions 2.32 and 3.05, and the more descriptive analyses by SPSS, version 22.

## Results

Table 1 shows the characteristics of the sample. The sex distribution was almost 50/50. The prevalence of use of ADHD medication in 2011 was 3.7%. The children are quite evenly distributed over the 50 urbanity levels.

**TABLE 1:** Characteristics of the sample at the level of the child (*n* = 248,270).

Characteristic	pct./mean ± *SD*
Sex: boys	51.4%
Age	8.6 ± 2.3
Prevalence of use of ADHD-medication in 2011	3.7%
Urbanity of neighborhood (based on address density)	
Very high	16.4%
High	23.8%
Moderate	20.2%
Low	20.3%
Not urban	19.3%
Average property value (in Euros)	
<145,000	11.2%
145,000–185,000	21.8%
185,000–225,000	24.5%
225,000–265,000	21.6%
265,000–305,000	10.4%
305,000–345,000	4.9%
>345,000	5.5%
Percentage of non-Western migrants (in 20 classes)	2.7 ± 2.9
Percentage of children < 15 years of age (in 20 classes)	4.3 ± 1.1
Percentage of green area within 250 m (in 20 classes)	7.8 ± 3.8
Percentage of green area within 500 m (in 20 classes)	9.2 ± 3.0
Average NDVI-score built-up area within 250 m (7 classes)	3.9 ± 1.7
Average NDVI-score built-up area within 500 m (7 classes)	3.9 ± 1.7

### Correlations between greenness indicators

Before regression analyses were performed, correlations between the different greenness indicators were calculated. The percentage of green area and the average NDVI score correlate *r* = 0.66 for the 250-m buffer and *r* = 0.67 for the 500-m buffer. This indicates residential environments with much green area also tend to have quite many smaller natural elements within the built-up part of the environment. However, the correlations are not that high that using both in the same regression analysis will cause multicollinearity problems. On the other hand, percentages for the 250- and 500-m buffers correlate with *r* = 0.90, and the average NDVI scores for those two distances *r* = 0.91. Thus, neither the two percentages nor the two NDVI scores can be used in the same analysis.

### Multilevel logistic regression analyses

The basic model, with only covariates, is presented in Table 2 (model 1). Boys have a higher prevalence of the use of ADHD medication than girls, and older children have a higher prevalence than younger children. Furthermore, the prevalence becomes lower with higher average property values for the neighborhood, as well as with increasing percentages of non-Western immigrants among the neighborhood population. On the other hand, the prevalence becomes higher with increasing percentage of children < 15 years in the neighborhood. Finally, in very highly urban neighborhoods, the prevalence is lower than in non-urban neighborhoods, while it is highest in moderately urban neighborhoods.

**TABLE 2:** Logistic regression models for prevalence of ADHD medication with interaction between percentage of green area within 250 m and average property value (in three categories); neighborhood as second level (*n* = 248,270).

	Odds ratio (95% confidence interval)		
	
	Model 1	Model 2	Model 3
Constant			***0.019 (0.017–0.022)***
Sex			
Boy	***3.511 (3.337, 3.695)***	***3.511 (3.337, 3.695)***	***3.511 (3.337, 3.695)***
Girl (ref.)	-	-	-
Age	***0.763 (0.755, 0.770)***	***0.763 (0.755, 0.770)***	***0.763 (0.755, 0.770)***
Avg. property value [joint Chi^2^ (df)]			***171.6 (6); p* < *0.001***
<145,000 (ref.)	–	–	–
145,000–185,000	0.969 (0.875, 1.072)	0.954 (0.860, 1.059)	0.928 (0.836, 1.029)
185,000–225,000	***0.829 (0.746, 0.922)***	***0.814 (0.732, 0.905)***	***0.796 (0.715, 0.887)***
225,000–265,000	***0.675 (0.604, 0.755)***	***0.665 (0.595, 0.744)***	***0.647 (0.577, 0.724)***
265,000–305,000	***0.594 (0.523, 0.675)***	***0.589 (0.518, 0.671)***	***0.570 (0.500, 0.650)***
305,000–345,000	***0.586 (0.500, 0.686)***	***0.589 (0.503, 0.691)***	***0.548 (0.463, 0.649)***
>345,000	***0.561 (0.484, 0.650)***	***0.567 (0.490, 0.657)***	***0.527 (0.449, 0.617)***
Pct. non-Western migrants (1–20)	***0.964 (0.949, 0.979)***	***0.965 (0.950, 0.980)***	***0.960 (0.945, 0.975)***
Pct. children < 15 (1–20)	***1.062 (1.033, 1.091)***	***1.063 (1.034, 1.092)***	***1.069 (1.040, 1.099)***
Urbanity of neighborhood [Joint Chi^2^ (df)]			***39.7 (4); p* < *0.001***
Very high	**0.844 (0.752, 0.947)**	***0.754 (0.661, 0.860)***	***0.761 (0.666, 0.870)***
High	*1.097 (1.011, 1.192)*	1.006 (0.914, 1.107)	1.018 (0.925, 1.121)
Moderate	**1.131 (1.044, 1.226)**	1.051 (0.961, 1.150)	1.062 (0.968, 1.164)
Low	1.023 (0.944, 1.109)	0.964 (0.882, 1.053)	0.971 (0.889, 1.061)
Non-urban (ref.)	–	–	–
Pct. green area 250 m (1–20)		***0.986 (0.978, 0.994)***	***0.970 (0.957, 0.984)***
Pct. green area × Avg. prop. value [Joint Chi^2^ (df)]			**10.9 (2); *p* < 0.01**
Pct green ×<185,000 (ref.)			–
Pct green × 185,000–305,000			**1.021 (1.005, 1.037)**
Pct green ×>305,000			**1.031 (1.011, 1.052)**
Variance at neighborhood level (standard error)	0.197 (0.016)	0.199 (0.016)	0.198 (0.016)

NB, percentages in 5% classes; all non-categorical variables centered beforehand.

Significance levels: italic, 0.05 level, bold, 0.01 level; italic and bold, 0.001 level.

The logistic regression analyses in which the greenness indicators for the 250-m buffer are added to the basic model (one by one) show that the percentage of green space is significantly associated with the prevalence of ADHD medication use, with the prevalence being lower when the percentage of green area is higher (Table 2, model 2). The average NDVI score for the built-up area is not significantly associated with the prevalence (OR = 0.988; 95% CI: 0.971–1.006). We also ran a model with both the percentage of green space and the average NDVI score for the built-up area included, checking that multicollinearity did not constitute a problem (VIF for percentage = 2.2, VIF for NDVI = 1.9). Also, when added after the percentage of green area is already included in the model, the predictive contribution of the average NDVI score for the built-up area within the 250-m buffer is not significant (OR = 1.002; 95% CI: 0.0983–1.022), whereas the parameter for the percentage of green area remains the same: OR = 0.986 (95% CI: 0.976–0.996; *p* < 0.01).

The regression results for the greenness indicators for 500-m buffer are quite similar to those for the 250-m buffer (not in table). Also, the parameter for the percentage of green area is significant, and the association is negative: OR = 0.985 (95% CI: 0.976–0.995; *p* < 0.01). The parameter for the average NDVI score of the built-up area within 500 m added to model 1 is not significant (OR = 0.989; 95% CI: 0.970–1.009), and neither it is significant when added to the model that already includes the percentage of green area (OR = 1.004; 95% CI: 0.983–1.026), whereas also the parameter for the percentage of green area stays virtually the same: OR = 0.984 (95% CI: 0.975–0.994); *p* < 0.01).

The analyses were repeated with family doctor as the second level, rather than neighborhood. The results were quite similar, with the same green space parameters being significant (not in table). The between variance for family doctor was somewhat smaller than that for neighborhood. For example, for the basic model (model 1), it was 0.140 (*SE* = 0.014).

### Additional analyses

Given the similar results for 250 and 500-m buffers, and neighborhood being a larger source of variation than family doctor, additional analyses were only performed for the 250-m green area percentage with neighborhood as the second level. First, we checked for non-linearity by adding a quadratic term for the percentage of green area (centered beforehand, added to model 2 in Table 2). This quadratic green area parameter was not significant (OR = 0.999; 95% CI: 0.997–1.001). Based on two earlier studies showing that the relationship between green space and ADHD-related behavior depended on SES (Balseviciene et al., 2014; Flouri et al., 2014), we explored moderation by SES. We tested for an interaction between the percentage of green space and the average residential property value. The results show that the interaction is significant (see Table 2, model 3). The negative relationship between green space and the prevalence of the use of ADHD medication is strongest in the neighborhoods with the lowest average residential property value and becomes weaker to non-existent when this property value rises. Following Markevych et al. (2014), we also explored moderation by sex using a separate model (i.e., instead of residential property value). The interaction between the percentage of green space and the sex of the child was not significant (OR = 0.998; 95% CI: 0.984–1.012). Also, the interaction between age and percentage of green space was not significant (OR = 1.001; 95% CI: 0.999–1.003).

The significant interaction between the percentage of green space and property values makes it of interest to look at the relationship between the presence of green space and the average residential property value within the neighborhood. The seven property value classes differ significantly (*p* < 0.001) in the amount of green area present. The relationship is predominantly linear in nature: the percentage of green area within 250 m increases with the property value (see Table 3). Translating the green area classes back to the original percentages, in the lowest residential property value class, the average percentage lies between 30 and 35%, whereas in the highest residential property value class, it lies between 45 and 50%, signifying an average difference in the green area percentage of at least 10% points.

**TABLE 3:** Amount of green area within 250 m by category of average of residential property value within the neighborhood (*n* = 248,270).

Category of residential property value (in euros)	Percentage of green space (in 20 5%-classes)	Standard deviation	Number of children
<145,000	6.8	4.2	27,838
145,000–185,000	7.0	2.9	54,218
185,000–225,000	7.4	3.2	60,823
225,000–265,000	7.9	3.5	53,653
265,000–305,000	8.7	4.3	25,924
305,000–345,000	9.8	5.2	12,048
>345,000	10.4	5.1	13,766
Total	7.8	3.8	248,270

## Discussion

The use of ADHD medication by children is negatively related to the amount of residential green space. This is the case for the percentage of green area within a buffer of 250 m and, to a similar extent, for that within a buffer of 500 m. The relationship differs by the average residential property value within the neighborhood. It is strongest in the category of lowest property value neighborhoods and non-existent in the category of highest property value neighborhoods. In the lowest property value neighborhoods (<145,000 Euro in 2012), a difference of 20% points of green space (25 vs. 45%) is associated with an over 10% lower probability of the child using ADHD medication. The observed beneficial association is in line with the outcomes of previous as well as more recent studies on green space and ADHD-related symptoms among children as reported by their parents/guardians and/or teachers, as well as with those of a study using a formal ADHD diagnosis as outcome measure (Markevych et al., 2018; Sakhvidi et al., 2022; Yuchi et al., 2022). It is also in line with the more general finding that there is a beneficial association between greenness exposure and the neuropsychological development and mental health of children (Luque-García et al., 2021). Less is known about the moderation of these associations by SES, which was observed in this study. Although (a proxy of) SES is usually included as a covariate, including it also as a moderator is not standard practice. A recent study that did look into this, using different measures for all three variables involved, did not observe such a moderating effect (Dzhambov et al., 2022). In fact, in that study, distance to nature in the residential environment was detrimentally associated with having behavioral problems.

Assuming causality for a moment, we briefly discuss the wider implications of a lower prevalence of ADHD. Le et al. (2014) estimated the societal costs in the Netherlands for children and adolescent to range between 9,860 and 14,483 Euro per case (2012 values). More recent U.S. figures are somewhat lower. According to Schein et al. (2022a), the societal economic burden of ADHD is US$ 6,799 per child annually. During adolescence, the burden is higher: US$ 8,349 per adolescent. In adulthood, the costs increase further to 14,092 per adult (Schein et al., 2022b). The latter is mainly of consequence of the negative impact of ADHD on long-term academic outcomes (Arnold et al., 2020), affecting earning capacity in adulthood. For example, in an U.S.-based study, children with formally diagnosed ADHD and receiving treatment, usually including medication, were estimated to earn even 1.27 million US$ less over their working lifetime than otherwise comparable individuals (Pelham et al., 2020). In Denmark, Jennum et al. (2020) also observed substantially lower earned incomes of people with ADHD after diagnosis (and presumably getting some form of treatment) than matched controls. Beyond these economic consequences, the quality of life of children diagnosed with ADHD is impaired, often also still in adulthood (Di Lorenzo et al., 2021; Faraone et al., 2021). Nigg et al. (2020) conclude that despite the availability of ever more sophisticated treatments, long-term outcomes are largely unchanged and deeply concerning. All in all, the societal costs of ADHD are substantial, making it worthwhile to consider investing in preventive measures. Increasing the amount of green space in poor neighborhoods with low levels of green space at present might be one way of prevention. Assessing the cost-to-benefit ratio of a 20% point increase in green area in deprived neighborhoods to achieve a 10% decrease in ADHD prevalence is beyond the scope of this article. However, it is important to note that urban greening is not only likely to beneficially affect ADHD prevalence but also that of other disorders and diseases (Maas et al., 2009). Furthermore, beyond generating health and wellbeing benefits, it may also contribute to climate change adaptation and urban biodiversity (Butt et al., 2018).

Given the cross-sectional nature of the study, the causality of this association is open to discussion. However, we did try to rule out likely alternative explanations by including several covariates in our statistical analyses, such as level of urbanity and average property values. The percentage of non-Western immigrants proved to be an important factor in this respect because it is negatively associated with both the average residential property value and the prevalence of use of ADHD medication, whereas the residential property value itself is also negatively associated with the prevalence of use. The relationship between ethnicity and the use of ADHD medication seems to be at least partly due to a cultural difference in the perception of the same type of ADHD-related behavior (Bevaart et al., 2012). It may be noted that to the extent that such behavior is indeed indicative of an actual disorder, affecting the quality of life of the child negatively, the present results may underestimate the relationship between green space and ADHD.

As for which type of green space is most likely to be beneficial, green elements within the residential environment outside green areas did not show a similar relationship with the prevalence of use of ADHD medication, neither when it was the only greenness indicator in the regression model nor when added after the percentage of green area was already included. Therefore, the presence of green areas seems to be more important than that of smaller elements such as street trees and domestic gardens. This might be taken as an indication that it is especially by outdoor play that the relationship occurs (see Amoly et al., 2014; Flouri et al., 2014), with (at least some) green areas offering attractive opportunities for this type of activity (see, e.g., Grigsby-Toussaint et al., 2011). According to Chaudhury et al. (2019), neighborhood public open spaces are preferred local destinations for children, especially as play areas (see also Brockman et al., 2011). In addition, they conclude that for autonomous play, unsupervised by parents, parents’ consent is important. To a large extent, this consent is based on the safety of the green area, as well as that of the route to that area, as perceived by parents (Qiu and Zhu, 2021; Visser and van Aalst, 2022). Furthermore, not only officially designated (green) playgrounds are likely to be relevant but also informal playgrounds (Visser and van Aalst, 2022), including undeveloped green areas, at least when trees are present (Janssen and Rosu, 2015). Furthermore, it is likely that such green areas do not need to be very large. Lachowycz et al. (2012) concluded that small green areas may be more important for outdoor play in this age category than (larger) parks. All in all, especially small (but not too small) nearby green areas that allow and afford play activities and are considered safe by parents (and children) may be relevant if the observed association is indeed mediated by time spent on outdoor play in such areas. Note that we do not mean to imply that it is (only) the physical activity associated with the outdoor play that is of importance. Also, the exposure to nature as such may play a role.

The pattern of the amount of nearby green space being stronger beneficially associated with the mental wellbeing of children living in less wealthy neighborhoods is consistent with the findings of Balseviciene et al. (2014) and Flouri et al. (2014). Also, it fits a more general pattern of beneficial associations between nearby green space and human health and wellbeing being stronger for less affluent people (Rigolon et al., 2021). At the same time, our additional analyses also showed that children living in less affluent neighborhoods tend to have less nearby green space. This finding is also consistent with the more generally observed pattern of people with a low SES having poorer access to green space (Schüle et al., 2019; De Vries et al., 2020). Differently speaking, those who are likely to benefit most from having green space nearby tend to have the least in their residential environment.

### Strengths and limitations of the study

A strength of the study is that it makes use of administrative data. This precludes a self-selection bias with regard to participating in the study. Another strength is that the data were available at the individual child, rather than only at a spatially aggregated level. Furthermore, the large number of children in the database made it possible to test more complex models, for example, with urbanity as a categorical covariate and an interaction between average residential property values and the percentage of green area. An additional advantage is that the study employs medication use as an indicator and thereby complements previous studies which have been largely based on (possibly quite subjective) ratings of the children’s behavior by their parents. This does not mean that the present study has no limitations. To begin with, as already mentioned, the children in the Achmea Health Database cannot be considered representative of all Dutch children. A more specific limitation in this regard is that only children who (a) are brought to the attention of the family doctor (or a pediatrician/other specialist), (b) are diagnosed with ADHD, and (c) are subsequently prescribed ADHD-related medication have been identified as suffering from ADHD. This was already acknowledged in the Introduction (see Figure 1). Starting with the last step in the chain (c), when a broad definition of ADHD is used (ICPC-codes P20, P21, P22), in 2012, 5.9% of the Dutch children aged between 0 and 17 years were registered as having ADHD by their family doctors (Prins and Van Dijk, 2015). Of these children, 25.5% were prescribed ADHD medication by the family doctors. Although that age range (0–17 years) is much wider than the one used here (5–12 years) and the ADHD prevalence differs by age, and that this type of medication may also have been prescribed by a specialist, the latter percentage strongly suggests that in the Netherlands, a considerable proportion of children diagnosed with ADHD do not get ADHD medication prescribed. Of the children with clinically diagnosed ADHD, those with more severe hyperactivity/impulsivity symptoms are more likely to be prescribed ADHD medication (Mowlem et al., 2019). To our knowledge, representative figures regarding the preceding two steps (a) and (b) are not available for the Netherlands. However, ethnicity was included as a confounder in our analyses because of an observed lower inclination of people with a non-Western ethnic background to seek medical assistance when a child displays ADHD-related behavior. These issues obviously affect the representativeness of our data with regard to all (Dutch) children with ADHD. However, given the steps needed to prescribe ADHD medication, with symptom severity playing an important role, the children who do get them prescribed are likely to constitute the more severe cases. One could argue that this makes the observed association between the percentage of green area and prevalence of use of ADHD medication even more interesting. Furthermore, if contact with nature reduces severe ADHD symptoms, it is not unlikely that children with less severe ADHD symptoms will also benefit from such contacts. Another limitation was that the Achmea Health Database contained limited information on the background characteristics of the children. For this reason, we used sociodemographic characteristics of the neighborhood relating to SES and ethnicity as proxies. It would be an improvement to (also) have information on such characteristics at the individual level of the child or the household.

Furthermore, as already mentioned, the study is cross-sectional in nature, limiting the ability to arrive at firm conclusions regarding the causality of the observed relationships. In addition to this, we also only looked at green space in the residential environment and did so in a static way (Helbich, 2018). During the course of the day, children may also move into other environments, for example, when attending school, making these environments relevant as well (see, e.g., Yang et al., 2019; Dzhambov et al., 2022). Furthermore, data on mediating factors, such as the use of green spaces for outdoor play, were not available. Such data would have helped assess the plausibility of a causal interpretation. Finally, given that contact with nature, mainly in the form of outdoor play, is assumed to be an important mediating factor, the green space indicator that was used is also quite crude. Not all green areas are suited for (autonomous) outdoor play. A “playability” qualification of green areas would bring more nuance in comparing residential neighborhoods (see also Janssen and Rosu, 2015).

Despite these limitations, we feel that this study adds to the evidence base that contact with nature is important for the health and wellbeing of children, especially those living in deprived neighborhoods.

## Data availability statement

The datasets presented in this article are not readily available because data can only be made available upon request and under certain conditions after approval by relevant Zilveren Kruis (formerly Achmea) Health Database governance bodies. Requests to access the datasets should be directed to corresponding author.

## Ethics statement

Ethical review and approval was not required for the study on human participants in accordance with the local legislation and institutional requirements. Written informed consent from the participants or their legal guardian/next of kin was not required to participate in this study in accordance with the national legislation and the institutional requirements.

## Author contributions

Both authors listed have made a substantial, direct, and intellectual contribution to the work, and approved it for publication.
